RETRACTED

# Deep Possibilistic *C*-means Clustering Algorithm on Medical Datasets

**DOI:** 10.1155/2022/3469979

**Published:** 2022-04-16

**Authors:** Yuxin Gu, Tongguang Ni, Yizhang Jiang

**Affiliations:** ^1^School of Artificial Intelligence and Computer Science, Jiangnan University, Wuxi, Jiangsu 214122, China; ^2^School of Computer Science and Artificial Intelligence, Changzhou University, Changzhou, Jiangsu 213164, China

## Abstract

In the past, the possibilistic *C*-means clustering algorithm (PCM) has proven its superiority on various medical datasets by overcoming the unstable clustering effect caused by both the hard division of traditional hard clustering models and the susceptibility of fuzzy *C*-means clustering algorithm (FCM) to noise. However, with the deep integration and development of the Internet of Things (IoT) as well as big data with the medical field, the width and height of medical datasets are growing bigger and bigger. In the face of high-dimensional and giant complex datasets, it is challenging for the PCM algorithm based on machine learning to extract valuable features from thousands of dimensions, which increases the computational complexity and useless time consumption and makes it difficult to avoid the quality problem of clustering. To this end, this paper proposes a deep possibilistic *C*-mean clustering algorithm (DPCM) that combines the traditional PCM algorithm with a special deep network called autoencoder. Taking advantage of the fact that the autoencoder can minimize the reconstruction loss and the PCM uses soft affiliation to facilitate gradient descent, DPCM allows deep neural networks and PCM's clustering centers to be optimized at the same time, so that it effectively improves the clustering efficiency and accuracy. Experiments on medical datasets with various dimensions demonstrate that this method has a better effect than traditional clustering methods, besides being able to overcome the interference of noise better.

## 1. Introduction

Clustering is an important way of data analysis and machine learning, using unsupervised learning methods. It splits a set of data into different clusters according to a specific division, which groups similar data into one cluster and divides unrelated data into different clusters. With the rapid advancement of artificial intelligence and the growing interest in the medical field in recent years, clustering has become increasingly used in medicine, [1, 2]. Clustering algorithms can reveal hidden information in medical data, which is useful for medical research and helps doctors with diagnosis. As one of these clustering algorithms, the possibility *C*-mean clustering method [3, 4] was initially proposed to overcome the sensitivity to noise and outliers caused by the normalization of affiliation in the fuzzy *C*-means clustering method (FCM) [5]. PCM relaxes the constraint in FCM that the sum of the affiliation of the sample points to the cluster centers equals 1 and takes into account the possibility that each sample point belongs to each cluster center. In that case, noises and outliers have little influence on the cluster center parameters during the iterative process, implying that noises may have little association with all cluster centers. Satisfactorily, the PCM algorithm is able to be well applied to medical image clustering [6]. However, it was also found by Barni et al. [7] that while PCM can reduce the effect of noise in the dataset to some extent, it also generates the problem of overlapping clustering centers due to neglecting the differentiation between the data clusters at the same time. In addition, the accuracy of the PCM algorithm is severely constrained by the parameters of the initialized clustering centers. To this end, Nikhil et al. proposed the fuzzy possibility *C*-means algorithm (FPCM) [8] improved by PCM, which considered both the fuzzy affiliation of FCM and the possibility concept of PCM, paying attention to both the differentiation between clusters and the dependence of each point on the cluster centers. However, while the FPCM method removes the row sum restriction, it also creates a column sum constraint for each cluster. As a result, Nikhil et al. introduced the PFCM algorithm, which removes PFCM's column sum restriction and combines the benefits of FCM, PCM, and FPCM to improve the clustering impact even further [9]. In response to the PCM algorithm which is easy to fall into the coincidence of cluster centers, Timm et al. advocated adding a cluster repulsion term that measures cluster-to-cluster exclusion to the PCM's objective function [10]. This objective function is optimal only when the distance between clusters and data within clusters is minimized and the distance between cluster centers is maximized.

RETRACTED

Despite the fact that the above-mentioned algorithms outperform some traditional machine learning-based clustering algorithms in small datasets, they are nonetheless overwhelmed when confronted with huge datasets with both sample size and dimensionality expansion. At this point, it is important to rely on effective dimensionality reduction and feature extraction means to deal with complex data for clustering purposes. Nowadays, the widely used dimension reduction tools comprise linear methods represented by principal component analysis (PCA) [11] and nonlinear methods represented by kernel methods [12], which have experimentally verified the feasibility of their combination with PCM. For example, the kernel possibility *C*-mean clustering proposed by Rhee et al. [13] applies the Gaussian kernel function to the PCM algorithm. The method with good clustering performance is applicable to not only spherical datasets but also nonspherical datasets and also inherits the advantage of PCM noise immunity. The above traditional dimensionality reduction methods, whether linear or nonlinear, all start by mapping high-dimensional data into a low-dimensional feature space and then perform the clustering operation. Although these methods reduce the computational complexity to a certain extent, since dimensionality reduction and clustering are two separate processes, the extracted features after dimensionality reduction may not be suitable for clustering. However, whether the extracted features are conducive to clustering is precisely the key factor that affects the effectiveness of clustering.

Over the past few years, deep neural networks (DNN) have been widely used in large-scale and deep-level feature extraction because of their powerful nonlinear mapping capability. Autoencoder (AE) [14] is a special type of DNN, which can be divided into two parts: encoder and decoder, where the former is used to reduce the dimension of the data, while the latter is used to reconstruct the feature representation in low-dimension space back to the original dimension. Its advantage is to minimize the reconstruction loss between the output data reconstructed by AE's decoder and the original data by iteratively training the network, thus obtaining a valid feature representation of the training sample. So far the autoencoder has now been combined with many traditional clustering methods and the feasibility of such combinations has been experimentally demonstrated. For instance, the deep embedding clustering model (DEC) proposed by Xie et al. [15] combines autoencoder and Kullback–Leibler (KL) divergence [16]. DEC first low-dimensionalises the data using the autoencoder and then calculates the probability matrix of the reduced-dimension data called soft assignment according to the *t*-distribution principle, which is used to calculate the KL scatter loss together with the author's proposed target auxiliary distributions. Yang et al. also proposed the deep clustering network (DCN) [17], which is the combination of the autoencoder with the *k*-means algorithm. Since the affiliation of the *K*-means algorithm is discrete and nonderivable, the parameters of the autoencoder and the parameters of the clustering center in this method can only be optimized in an alternating manner. It was later improved by the deep *k*-means algorithm (DKM) [18], which further improved the clustering effect by making the clustering loss of *k*-means derivable through the softmax function. DKM allows simultaneous optimization of the autoencoder and clustering centers.

RETRACTED

Although the DKM makes use of a differentiable *k*-means method via the softmax function, which allows it to participate in the iterative optimization process simultaneously with the autoencoder, it is clear that using this optimized *K*-means algorithm is more complex than the naturally differentiable soft-partition clustering algorithms like FCM and PCM. Given that the PCM algorithm has some antinoise performance when compared to other soft-partition clustering algorithms, we use a combination of autoencoder and PCM algorithm called DPCM in this paper. This algorithm takes advantage of both PCM for gradient descent and deep neural networks for feature extraction of large-scale high-dimensional datasets. The work done in this paper is as follows:

1. Combine the deep neural network with the possibilistic *C*-means method: DPCM uses the encoding part of the autoencoder to reduce the datasets' dimension and performs PCM clustering on the feature representation generated after the dimensionality reduction. Because of the PCM's continually derivable nature, it is possible to update network parameters and clustering centers at the same time. For high-dimensional datasets, the method effectively improves the clustering effect
2. Extensive experimentation and validation: to validate the flexibility of the method on different medical datasets, we conducted extensive comparative experiments on medical datasets of various sample sizes and dimensions. The experiments demonstrate that the method is highly feasible for medical image clustering, and its accuracy is not limited to large datasets with inflated dimensionality and sample size
3. Demonstrates excellent noise immunity: we conducted comparison experiments between the dataset with the addition of the Gaussian noise at the ratio of 1% and 3% and the original dataset, respectively, to verify whether the present method inherits the noise resistance ability of the PCM algorithm. The experiments show that to a certain extent, the clustering effect and accuracy of DPCM are less affected by noise interference than other methods. It is possible to say that DPCM has some noise immunity

We organize the rest of this paper as follows. Firstly, related work is reviewed in Section 2. The proposed method DPCM is introduced in Section 3. The results of comparison experiment are shown in Section 4. Finally, conclusions and future work exploration are summarized in Section 5.

RETRACTED

## 2. Related Work

### 2.1. FCM

For a given dataset *X* = {*x*_1_, x_2_, ⋯, *x*_*N*_}, letting the clustering center be {*v*_1_, *v*_2_, ⋯, *v*_*K*_}, *u*_*ij*_ is denoted, and the probability estimates how much of that the sample *x*_*j*_ belongs to the cluster center *c*_*i*_, where the value needs to satisfy

(1) $$\begin{array}{c} 0\leq u_{ij}\leq 1,\overset{K}{\underset{i=1}{\sum }}\;u_{ij}=1. \end{array}$$

Thus, the membership matrix is expressed as *U* = {*u*_*ij*_|1 ≤ *i* ≤ *K*, 1 ≤ *j* ≤ *N*}; *m* is a constant larger than 1. It is known that when we get

(2) $$\begin{array}{c} \begin{array}{c} \underset{V,U}{\min}\;\left(J_{\text{FCM}}\left(V,U\right)=\overset{K}{\underset{i=1}{\sum }}\;\overset{N}{\underset{j=1}{\sum }}\;u_{ij}^{m}{||x_{j}-v_{i}||}^{2}\right)\\ \; \end{array}, \end{array}$$

it must meet. For each cluster center, the distance from the sample inside the cluster to this cluster center is the smallest, and it is less than the distance from these samples to other clusters. Considering the range of values of *u*_*ij*_, the objective function can be defined as

(3) $$\begin{array}{c} \left.F=J_{\text{FCM}}\left(V,U\right)=\overset{K}{\underset{i=1}{\sum }}\;\overset{N}{\underset{j=1}{\sum }}\;u_{ij}^{m}{||x_{j}-v_{i}||}^{2}\right)+\lambda \left(1\overset{K}{\underset{i=1}{\sum }}\;u_{ij}\right). \end{array}$$

Respectively, setting *∂F*/*∂u*_*ij*_ = 0 and *∂F*/*∂v*_*i*_ = 0, the iterative paths of *u*_*ij*_ and *v*_*i*_ are as follows:

(4) $$\begin{array}{c} u_{ij}=\frac{1}{\sum_{k=1}^{K}\;{\left(||x_{j}-v_{i}||/||x_{j}-v_{k}||\right)}^{2/\left(m-1\right)}},\;\;i=1,2,\cdots K;\text{j}=1,2,\cdots ,N, \end{array}$$

(5) $$\begin{array}{c} v_{i}=\frac{\sum_{j=1}^{N}\;u_{ij}^{m}x_{j}}{\sum_{j=1}^{N}\;u_{ij}^{m}},\;i=1,2,\cdots ,K. \end{array}$$

Equations (4) and (5) will iterate repeatedly until the algorithm converges.

### 2.2. PCM

The PCM algorithm liberalizes the constraint that the sum of affiliation of a sample point to all clustering centers is 1 in FCM and proposes a new concept of probability, using *u*_*ij*_ to denote the probability that the sample *x*_*j*_ is classified into the *i*-th cluster, taking the following range of values:

(6) $$\begin{array}{c} u_{ij}\in \left[0,1\right],0<\overset{n}{\underset{i=1}{\sum }}\;u_{ij}\leq n,\max_{i}\;u_{ij}>0. \end{array}$$

Therefore, the objective function is set to

(7) $$\begin{array}{c} J_{m}\left(U,V\right)=\overset{K}{\underset{i=1}{\sum }}\;\overset{N}{\underset{j=1}{\sum }}\;u_{ij}^{m}{||x_{j}-v_{i}||}^{2}+\overset{K}{\underset{i=1}{\sum }}\;\eta_{i}\overset{N}{\underset{j=1}{\sum }}\;{\left(1-u_{ij}\right)}^{m}. \end{array}$$

The parameter iteration paths are as follows:

(8) $$\begin{array}{c} v_{i}=\frac{\sum_{j=1}^{N}\;u_{ij}^{m}x_{j}}{\sum_{j=1}^{N}\;u_{ij}^{m}},\\ u_{ij}=\frac{1}{\left(1+{\left(d_{ij}/\eta_{i}\right)}^{1/\left(m-1\right)}\right)},\\ \eta_{i}=\frac{\sum_{j=1}^{n}\;u_{ij}^{m}d_{ij}}{\sum_{j=1}^{n}\;u_{ij}^{m}}, \end{array}$$

where the initial value of *η*_*i*_ needs to be set manually. The common practice is to first cluster the samples using the FCM algorithm and substitute the parameters of the cluster centers obtained after clustering into the formula to obtain the initial value of *η*_*i*_. It is also possible to simply calculate the value of *η*_*i*_ from the parameters of randomly selected clustering centers, but the clustering results obtained in this way are often less stable than the former.

RETRACTED

### 2.3. Autoencoder

The autoencoder (AE) is a powerful unsupervised learning method consisting of two parts, the encoder and the decoder, which are symmetrically structured [19]. The two components are repeatedly optimized until the minimum reconstruction error is obtained, thus extracting the most representative set of features from the complex data.

Suppose that there are *n* samples in the dataset to be handled, and *ϕ*()  and *φ*() are the functions used for the encoding and decoding processes separately; if we use the mean square error to measure the error between the reconstructed samples of the AE and the original input samples, the reconstructed loss function of this AE will be expressed as

(9) $$\begin{array}{c} \;L_{\text{rec}}=\frac{1}{N}\overset{N}{\underset{i=1}{\sum }}\;{||x_{i}-\varphi \left(\phi \left(x_{i}\right)\right)||}^{2}. \end{array}$$

The optimization objective of the AE is to obtain the network parameters that minimize this reconstruction error:

(10) $$\begin{array}{c} \phi ,\varphi =\arg\min_{\phi ,\varphi }\;L_{\text{rec}}. \end{array}$$

## 3. Deep Possibilistic *C*-means Clustering

Instead of using the *K*-means algorithm in DCN, which is not suitable for simultaneous iterative optimization with the deep neural network (DNN), DPCM adopts the PCM algorithm using soft affiliation naturally that is capable of updating parameters by stochastic gradient descent (SGD) with AE synchronously. The DPCM algorithm combines AE with the traditional PCM algorithm, optimizing both the clustering loss generated from PCM and the reconstruction loss based on the autoencoder. Specifically, the network is defined as shown in Figure 1, where *C* denotes all the parameters of the clustering centers generated by each iteration, as *Ɵ* denotes all the parameters generated during the autoencoder iteration, both of which can be gradient descended simultaneously.

RETRACTED

In the deep PCM model, the sample *X* is dimensioned down through layer after layer to obtain feature representation as *ϕ*(X), which is further passed through the decoding part of AE to generate the reconstructed sample *X*′ = *φ*(*ϕ*(*X*)). Suppose the sample size is *N*. If we use the mean square error to measure the difference between the reconstructed samples and original samples, the loss of the AE component is specified as follows:

(11) $$\begin{array}{c} \text{AE}\_\text{loss}=\overset{N}{\underset{i=1}{\sum }}\;{||x_{i}-\varphi \left(\phi \left(x_{i}\right)\right)||}^{2}, \end{array}$$

where *ϕ*() denotes the function used by AE for the encoding part and *φ*() denotes the function used for the decoding part.

When the original dataset *X* is reduced to *W* dimensions in AE, *x*_*i*_ denotes the *i*-th sample data and *c*_*j*_ denotes the cluster center of the *j*-th cluster; then, *ϕ*(*x*_*i*_) denotes the feature representation of the sample *x*_*i*_ after the reduction to *W* dimensions, where *ϕ*(*x*_*i*_)_*w*_ is the value of the *w*-th feature of *ϕ*(*x*_*i*_) and *c*_*jw*_ is the value of the *w*-th feature of the *j*-th cluster center. Then, the distance of the sample *x*_*i*_ after dimensionality reduction from the computed clustering center *c*_*j*_ can be expressed as

(12) $$\begin{array}{c} d\left(\phi \left(x_{i}\right),c_{j}\right)=\overset{W}{\underset{w=1}{\sum }}\;{\left(\phi {\left(x_{i}\right)}_{w}-c_{jw}\right)}^{2}={||\phi \left(x_{i}\right)-c_{j}||}^{2}. \end{array}$$

The probability *u*_*ij*_ that the sample *x*_*i*_ in low-dimensional space belongs to the clustering center *c*_*j*_ can be expressed as

(13) $$\begin{array}{c} u_{ij}=\frac{{\left(1/||\phi \left(x_{i}\right)-c_{j}||\right)}^{2/\left(m-1\right)}}{\sum_{k=1}^{K}\;{\left(1/||\phi \left(x_{i}\right)-c_{k}||\right)}^{2/\left(m-1\right)}}=\frac{1}{\sum_{k=1}^{K}\left(\begin{array}{c} ||\phi \left(x_{i}\right)-c_{j}||\\ ||\phi \left(x_{i}\right)-c_{k}|| \end{array}\right)\;\left(2/\left(m-1\right)\right)}, \end{array}$$

where *m* is an artificially set value greater than 1 which is used to weight the affiliation.

Then, the clustering loss of PCM can be obtained as

(14) $$\begin{array}{c} \text{PC}{\text{M}}_{-}\text{loss}=\overset{N}{\underset{i=1}{\sum }}\;\overset{K}{\underset{j=1}{\sum }}\;u_{ij}^{m}d\left(\phi \left(x_{i}\right),c_{j}\right)=\overset{N}{\underset{i=1}{\sum }}\;\overset{K}{\underset{j=1}{\sum }}\;\frac{{||\phi \left(x_{i}\right)-c_{j}||}^{2}}{{\left(\sum_{k=1}^{K}\;{\left(||\phi \left(x_{i}\right)-c_{j}||/||\phi \left(x_{i}\right)-c_{k}||\right)}^{\left(2/\left(m-1\right)\right)}\right)}^{m}}. \end{array}$$

Sum the AE loss and the PCM loss with weights and we can get the objective function of this DPCM algorithm:

(15) $$\begin{array}{c} {\mathrm{Min}}_{\theta ,C}\;L=\min_{\theta ,C}\;\left(\text{A}{\text{E}}_{-}\text{loss}+\text{FC}{\text{M}}_{-}\text{loss}\right)=\min_{\theta ,C}\left(\;\overset{N}{\underset{i=1}{\sum }}{||x_{i}-\varphi \left(\phi \left(x_{i}\right)\right)||}^{2}+\overset{N}{\underset{i=1}{\sum }}\overset{K}{\underset{j=1}{\sum }}\;\frac{{||\phi \left(x_{i}\right)-c_{j}||}^{2}}{{\left(\sum_{k=1}^{K}{\left(||\phi \left(x_{i}\right)-c_{j}||/||\phi \left(x_{i}\right)-c_{k}||\right)}^{\left(2/\left(m-1\right)\right)}\right)}^{m}}\right), \end{array}$$

where *θ* denotes all the parameters of the AE and *C* denotes all the clustering centers.  Algorithm 1 gives the specific steps of the DPCM algorithm, where *m* is a parameter that needs to be set manually in the PCM algorithm.

RETRACTED

## 4. Experiment

In order to verify the effectiveness of the DPCM algorithm proposed in this paper and its practicality on medical datasets, we have done extensive experiments comparing the DPCM algorithm with five other clustering algorithms on medical image datasets, which are PCM, FCM, AGglomerative NESting (AGNES) [20], K-means++ [21], and K-medoids [22]. And we also added Gaussian noise with proportions of 1% and 3% for each dataset to verify the noise immunity performance of these six different clustering methods. All algorithms are implemented by using MATLAB R2019b.

### 4.1. Dataset

To verify the flexibility and adaptability of the DPCM algorithm in clustering medical datasets of different dimensions and sizes compared to traditional clustering algorithms, we used three 2D datasets with 28∗28 pixels and two 3D datasets with 28∗28∗28 pixels, respectively, from MedMNIST v2 [23] for testing. The five datasets are OrganAMNIST(2D), OrganCMNIST(2D), OrganSMNIST(2D), Adrenalmnist3D(3D), and FractureMNIST3D (3D).

Among them, Organ{A, C, S}MNIST are 3D CT images based on the liver tumor segmentation benchmark(LiTS)^25^, which have 784-dimensional data width and 11 labels for clustering and classification tasks. These datasets differ in viewpoint, cropped from the center slice of the 3D bounding box in the axial/coronal/sagittal view (planar), respectively. The sample sizes are 58850, 23660, and 25221, correspondingly.

The data width of Adrenalmnist3D (3D) and FractureMNIST3D (3D) are both 21952 with 2 and 3 labels, respectively. And the number of samples is 1743 and 1370, correspondingly.

### 4.2. Parameter Setting

#### 4.2.1. The Weighting Index *M*

In the FCM, PCM, and DPCM algorithm, we need to specify the weighting index *m* whose value is closely related to the effect of clustering. Therefore, we have done a lot of experiments on the value of *m* in each experiment, increasing gradually from 1.1 to 5.0. The experimental results show that for the five datasets used in this paper, *m* tends to achieve the best performance for the mentioned three clustering algorithms when its value is taken in the range of 1.2-2.0. However, in the Adrenalmnist3D dataset, the performance of the FCM algorithm does not change no matter how *m* is taken in the range of 1.2 to 2.0. Therefore, in this paper, we also gradually increase the value of *m* in the range of 2.0-5.0 at a pace of 0.5 and in the range of 5.0-10.0 at a pace of 1.0. Experimentally, we prove that in this dataset, whatever value of *m* is taken does not affect the FCM. The trend of the clustering effect of FCM, PCM, and DPCM with the change of *m* value is shown in Figure 2.

RETRACTED

#### 4.2.2. *K*-means++ and *K*-medoids

Only the parameter *k* needs to be set as the number of clusters of the dataset, where its values in OrganAMNIST, OrganCMNIST, OrganSMNIST, Adrenalmnist3D, and FractureMNIST3D are set to 11, 11, 11, 2, and 3, separately.

#### 4.2.3. FCM

*k* is the number of clusters. The weighting index *m* is set as 4.2.1. In addition, we need to set two parameters maxiter as 1000 and *ε* as 0.005 for terminating the iterative optimization of the program. Therefore, the iteration will come to an end right away when any of the following conditions are met: (1) the number of iterations is equal to the maxiter and (2) ||*U*^(*t*)^ − *U*^(*t* − 1)^|| < *ε*.

#### 4.2.4. PCM

The required parameters and values are the same as FCM. In addition, the initial value of the clustering centers is determined by the FCM after optimization.

#### 4.2.5. DPCM

The number of clustering centers *k* is set the same as Section 4.2.2. The weighting index *m* is set the same as Section 4.2.1.

### 4.3. Result Analysis

In this paper, the results of this experiment are evaluated using two external evaluation indicators commonly used in unsupervised cluster analysis, ACC [24] and NMI [25], where ACC denotes clustering accuracy and NMI denotes normalized mutual information, both of which take values ranging from 0 to 1. The higher these two values hold, the better the clustering effect shows. The expressions for ACC and NMI are specified as follows:

(16) $$\begin{array}{c} \text{NMI}\left(\Omega ,C\right)=\frac{I\left(\Omega ;C\right)}{\left(H\left(\Omega \right)+H\left(C\right)\right)/2},\\ \text{ACC}\left(C,S\right)=\max_{\psi }\;\frac{1}{N}\overset{N}{\underset{i=1}{\sum }}\;\chi \left\{s_{i}=\psi \left(c_{i}\right)\right\}, \end{array}$$

where *I*(*Ω*, C) denotes the interaction information between *Ω* and *C*, and it is expressed as follows:

(17) $$\begin{array}{c} I\left(\Omega ,C\right)=\underset{k}{\sum }\;\underset{j}{\sum }\;P\left(w_{k}\cap c_{j}\right)\log\frac{P\left(w_{k}\cap c_{j}\right)}{P\left(w_{k}\right)P\left(c_{j}\right)}=\underset{k}{\sum }\;\underset{j}{\sum }\;\frac{\left|w_{k}\cap c_{j}\right|}{N}\log\frac{N\left|w_{k}\cap c_{j}\right|}{\left|w_{k}\right|\left|c_{j}\right|},\\ H\left(\Omega \right)=-\underset{k}{\sum }\;P\left(w_{k}\right)\log P\left(w_{k}\right)=-\underset{k}{\sum }\;\frac{\left|w_{k}\right|}{N}\log\frac{\left|w_{k}\right|}{N}, \end{array}$$

where *P*(*w*_*k*_) denotes the possibility that *x* belongs to the cluster *w*_*k*_; *P*(*w*_*k*_∩*c*_*j*_) denotes the probability that *x* belongs to both sets *w*_*k*_ and *c*_*j*_.

RETRACTED

From the above two evaluation index criteria, as shown in Figure 2, the DPCM algorithm proposed in this paper is significantly more effective than other traditional clustering algorithms in clustering both the 784-dimensional 2D dataset and the 3D dataset with data dimension up to 21952.  Table 1 shows the results of ACC and NMI obtained by clustering DPCM with five other clustering algorithms on different datasets. The DPCM algorithm apparently greatly improves the clustering effect of the PCM algorithm. It can be seen that the deep PCM algorithm proposed in this paper can well combine the PCM with the autoencoder to maximize the clustering performance of the PCM algorithm and the dimensionality reduction advantage of the autoencoder, jointly promoting the advantages of each other.

### 4.4. Antinoise Performance

In order to verify whether the DPCM algorithm inherits the advantage of the PCM algorithm's strong noise immunity, we added Gaussian noise with proportions of 1% and 3% to each dataset and compared the experimental results with the original dataset to observe how ACC and NMI changed (the mean value of Gaussian noise is set to 0, and the variance is set to 0.05).

The performance comparison before and after adding noise can be seen in Tables 2–5. From the experimental results, we can easily see that in the case of adding 1% and 3% Gaussian noise, the ACC and NMI after DPCM clustering are better than other algorithms in ORGAN-A, ORGAN-C, AND ORGAN-S datasets; in the FRACTURE dataset containing 1% and 3% noise, DPCM still outperforms other algorithms in NMI, while the results of ACC are inferior to those of other algorithms; in the ADRENAL dataset with 1% and 3% noise, DPCM still outperformed the other algorithms in ACC, while NMI was inferior to the other algorithms. Since the first three datasets have in common that they are all 784-dimensional, on the other hand, the last two datasets are all 21952-dimensional. Therefore, we cannot rule out the possibility that the noise immunity of the DPCM will be affected by the dimensionality. However, in most cases, the DPCM algorithm not only outperforms the other algorithms in terms of the clustering effect but even slightly improves the results compared to the original datasets, so we can assume that DPCM has some noise immunity which is inherited from the PCM algorithm.

RETRACTED

## 5. Conclusion

In this paper, to further explore the potential of deep neural networks for clustering medical images, we combine the autoencoder with the soft-partition clustering method PCM. Since PCM uses the probability concept that can perform stochastic gradient descent instead of the discrete affiliation of *K*-means, the optimization of the clustering parameters can be performed together with the network optimization of AE. Therefore, the autoencoder is gradually iteratively optimized in the direction favorable to PCM clustering, which further improves the clustering efficiency and accuracy. We also found that the clustering performance of DPCM is higher than other clustering methods in the presence of 1%-3% Gaussian noise in the datasets, which proves that the DPCM algorithm has a certain resistance to noise interference, which makes it more adaptable. However, during the experiments, we also found that the improvement of the clustering effect of DPCM compared with traditional clustering methods did not show significantly on some datasets, which may be related to the adaptability of the network model or the selection of initial parameters. We should continue to pay attention to this aspect in the future.

## Figures and Tables

**Figure 1:** The structure of DPCM.

**Figure 2:** Trend of ACC and NMI of FCM, PCM, and DPCM under different values of *m*.

**Algorithm 1:** Deep possibilistic *C*-means algorithm.

**Table 1:** The results of ACC and NMI obtained by clustering DPCM with five other clustering algorithms on different datasets.

	KM	FCM	PCM	*K*-medoids	AGNES	Deep PCM
OrganA	ACC 0.571	0.459	0.401	0.176	0.589	0.608
	NMI 0.612	0.494	0.397	0.058	0.693	0.703
OrganC	ACC 0.488	0.542	0.383	0.17	0.516	0.625
	NMI 0.596	0.552	0.405	0.045	0.665	0.691
OrganS	ACC 0.436	0.372	0.377	0.166	0.465	0.502
	NMI 0.511	0.433	0.368	0.049	0.592	0.605
Fracture3D	ACC 0.388	0.397	0.426	0.41	0.388	0.448
	NMI 0.018	0.018	0.024	0.008	0.016	0.061
Adrenal3D	ACC 0.552	0.561	0.612	0.52	0.582	0.776
	NMI 0.023	0.025	0.029	0.003	0.032	0.038

**Table 2:** ACC performance on datasets with 1% Gaussian noise.

1% ACC	KM	FCM	PCM	*K*-medoids	AGNES	DPCM
OrganA	0.571	0.459	0.401	0.176	0.589	0.608
1% noise	0.560	0.460	0.406	0.178	0.542	0.607
OrganC	0.488	0.542	0.383	0.17	0.516	0.625
1% noise	0.488	0.533	0.381	0.17	0.521	0.626
OrganS	0.436	0.372	0.377	0.166	0.465	0.502
1% noise	0.436	0.371	0.377	0.167	0.451	0.507
Fracture	0.388	0.397	0.426	0.41	0.388	0.448
1% noise	0.398	0.390	0.425	0.41	0.398	0.412
ADRENAL	0.552	0.561	0.612	0.52	0.582	0.776
1% noise	0.556	0.561	0.612	0.55	0.581	0.776

RETRACTED

**Table 3:** NMI performance on datasets with 1% Gaussian noise.

	KM	FCM	PCM	*K*-medoids	AGNES	DPCM
OrganA	0.612	0.494	0.397	0.058	0.693	0.703
1% noise	0.607	0.496	0.406	0.076	0.684	0.712
OrganC	0.596	0.552	0.405	0.045	0.665	0.691
1% noise	0.596	0.551	0.435	0.039	0.653	0.697
OrganS	0.511	0.433	0.368	0.049	0.592	0.605
1% noise	0.513	0.435	0.370	0.048	0.582	0.609
Fracture	0.018	0.018	0.024	0.008	0.016	0.061
1% noise	0.016	0.020	0.028	0.018	0.022	0.036
ADRENAL	0.023	0.025	0.029	0.003	0.032	0.038
1% noise	0.024	0.025	0.031	0.006	0.032	0.027

**Table 4:** ACC performance on datasets with 3% Gaussian noise.

	KM	FCM	PCM	*K*-medoids	AGNES	DPCM
OrganA	0.571	0.459	0.401	0.176	0.589	0.608
3% noise	0.581	0.460	0.397	0.174	0.562	0.614
OrganC	0.488	0.542	0.383	0.17	0.516	0.625
3% noise	0.491	0.553	0.384	0.167	0.507	0.637
OrganS	0.436	0.372,	0.377	0.166	0.465	0.502
3% noise	0.435	0.372	0.379	0.166	0.456	0.515
Fracture	0.388	0.397	0.426	0.41	0.388	0.448
3% noise	0.387	0.397	0.429	0.408	0.408	0.424
ADRENAL	0.552	0.561	0.612	0.52	0.582	0.776
3% noise	0.551	0.563	0.588	0.551	0.580	0.776

**Table 5:** NMI performance on datasets with 3% Gaussian noise.

	KM	FCM	PCM	*K*-medoids	AGNES	DPCM
OrganA	0.612	0.494	0.397	0.058	0.693	0.703
3% noise	0.621	0.497	0.410	0.051	0.675	0.708
OrganC	0.596	0.552	0.405	0.045	0.665	0.691
3% noise	0.595	0.557	0.433	0.047	0.661	0.698
OrganS	0.511	0.433	0.368	0.049	0.592	0.605
3% noise	0.511	0.434	0.395	0.048	0.599	0.612
Fracture	0.018	0.018	0.024	0.008	0.016	0.061
3% noise	0.018	0.021	0.029	0.017	0.002	0.038
ADRENAL	0.023	0.025	0.029	0.003	0.032	0.038
3% noise	0.022	0.026	0.031	0.007	0.031	0.024

## Data Availability

The dataset used to support the findings of this study are available from the corresponding author upon request.
